# Design of Motion Detection Device in Sports Based on Deep Learning of Internet of Things

**DOI:** 10.1155/2022/2613318

**Published:** 2022-02-23

**Authors:** Shaolong Li, Changlei Zhou

**Affiliations:** ^1^Sports Reform and Development Research Center, Henan University School of Physical Education and Sport, Kaifeng 475001, Henan, China; ^2^College of Sports and Health, Linyi University, Linyi 276000, Shandong, China; ^3^Department of Leisure Services and Sports, Pai Chai University, Daejeon 35345, Republic of Korea

## Abstract

With the improvement of people's income levels in recent years, people have gradually begun to pay more attention to health, and the number of exercise and fitness people has increased year by year. People are gradually willing to pay for sports and fitness, increase sports consumption, and promote the development of the sports and fitness industry. This article aims to study the deep learning based on the Internet of things to make people aware of the importance of sports. Not loving sports is a major problem that contemporary people need to overcome. This article proposes how to design a motion detection device in sports based on deep learning of the Internet of things. Based on the calculation of the economic volume of the deep learning of the Internet of things and the questionnaire survey method, it can be seen that, in today's globalization, although everyone knows the importance of sports, they are unwilling to practice it and would rather spend more time on the Internet. The experimental results of this article show that more than 50% of college students are very interested in sports and fitness, but the actual use is less than 30%, which is not optimistic. In social surveys, this number will be even lower, with only 14% of people interested in sports. Big data is like a “double-edged sword.” It not only displays the user's exercise data in front of everyone through the built-in sensors of the mobile phone, but also manages their physical condition through these. How to use the strengths of sports applications at the same time properly disposing of private information is a part of the next development of sports applications that must be faced.

## 1. Introduction

In today's society, various communication means and technologies are constantly updated and developed. At the same time, the development of the network also moves from the Internet to the direction that all devices and machines can be connected to each other. The Internet of things (IOT) can be said to be an important part of the new generation of information technology. It has finally realized the interconnection among objects and people. In the past few years, deep learning has been regarded as one of the most popular methods in machine learning. Using deep learning theory to detect moving targets is an important application of mechanical learning in computer vision. The emergence of sports applications perfectly realizes the combination of the two. Whether the digitization of individual sports behavior will promote health behavior is also a new research direction in the field of health communication. However, scholars, Coleman, and others have conducted a large number of empirical studies on Internet sports and concluded that there is a phenomenon of system disconnection between online actions and offline action, which will enable users to label them with “lazy Activism” self-presentation behavior in the process of use. Teenagers are the main groups that the state focuses on participating in sports activities to improve their physical quality, and all countries also pay increasing attention to the development of the Internet of things. Therefore, it has inspired increasingly researchers to study the target tracking task. Moving object detection has become a hot topic in the field of computer vision. How to design a motion detection device in sports based on deep learning of Internet of things has become a difficult problem. The physical fitness test is to enable one to grasp and understand their physical condition and have a full understanding of one's own body to achieve the goal of health.

In today's era, the development of network information technology is very fast, and its application fields are becoming increasingly extensive. Network information has become an important part of the information society. Of course, we human beings have also entered a new network era. Information network has a large application field, and its service object range is further expanding. The Internet of things should be regarded as such a network, which can combine the Internet with a large number of goods and complete the communication between them, and finally complete the unified identification, positioning, monitoring, and management of goods. By studying the communication mode of sports application and exploring how sports application affects college students' healthy living habits, it can not only make college students pay more attention to their own health status, but also promote college students to increase sports and improve their physique. With the professional and market-oriented development of competitive sports, it has promoted the promotion of athlete communication. It puts forward higher requirements for the flow speed of athletes in post, industries, and regions. This kind of communication is the objective demand of social production and scientific integration. It is a spatial dynamic adjustment in accordance with the development law of athletes and the requirements of the social market. The exchange of athletes has promoted the pace of international development of competitive sports and played a positive role in the optimization of competitive sports talent resources in various countries and the rational allocation of regional talents.

Traditional social and community ties have declined as a result of increased geographical mobility, industrialization, and other factors. On the contrary, sports audiences continue to flourish. D. Travis believes that strong identification with a specific sports team can buffer depression and alienation. The position of the Academy of Nutrition, the Canadian Dietitian (DC), and the American Academy of Sports medicine (ACSM) is that carefully selected nutrition can improve the performance of sports activities and recovery strategies. These organizations provide guidelines for the appropriate type, amount, and timing of food, fluids, and supplements to promote optimal health and performance in different training and competitive sports scenarios. This position paper is prepared for members of the college, DC and ACSM, other professional associations, government agencies, industry, and the public [1]. Thevis M believes that, for nearly a century, large-scale college sports have always been a popular but problematic part of American higher education. Its challenges to traditional academic values have been recognized from the beginning, but in recent decades, these challenges have become more ominous as cable TV has become ubiquitous, and business opportunities and sports budgets have surged. In the second edition of his influential important Sports in American Universities, Klottfeldt continued to study the role of sports in American universities. Based on his argument, commercial sports have become the core function of universities engaged in sports [2]. Hao pointed out that deep learning is a branch of machine learning. It attempts to use multilayer neurons composed of complex structures or nonlinear transformations to model the high-level abstraction of data. Hao pointed out that deep learning is a branch of machine learning that uses multiple layers of neurons composed of complex structures or nonlinear transformations to simulate high-level abstraction of data. With the increase of data and computing power, neural networks with more complex structure have attracted extensive attention and been applied to various fields. This paper summarizes the deep learning in neural networks, including popular architecture models, and training algorithms [3]. Levine explains the coordination method of hand and eye, which is the learning basis of monocular image capturing robot. To learn the coordination of hand and eyes, a large-scale convolutional neural network is trained. Only single lens camera images are used, which is independent of camera calibration and current. The probability that the action of the gripper task space is connected with normal grasping is predicted. This requires the network to observe the spatial relationship between the handle and the objects in the scene and learn the coordination between the hand and the eye. Then, the network real-time servo gripper is used to make the clamping successfully. The experimental evaluation of Levine shows that Levine method can realize effective real-time control, correctly grasp new objects and correct errors through continuous servo [4]. Classification is one of the hottest topics in hyperspectral remote sensing. In the past 20 years, Song and Brandt-Pearce has proposed many methods to deal with hyperspectral data classification. However, most of these do not extract deep features within the layer. This article introduces the concept of deep learning on the Internet. Firstly, according to the classical classification based on spectral information, the adaptability of the stacked automatic encoder is verified. Second, a new method of classification using spatial advantage information is proposed. Song and Brandt-Pearce proposed a new deep learning framework, which can combine these two functions to obtain the highest classification accuracy. The framework combines principal component analysis (PCA), deep learning architecture, and logistic regression. Specifically, as a deep learning architecture, stacked automatic encoder aims to obtain useful advanced features [5], a printable, multifunctional, flexible, and removable patch for health monitoring with human motion detection function. Real-time health care monitoring can predict and prevent disease or improve treatment by early diagnosis of disease. Wearable and comfortable sensing devices are needed to continuously monitor a person's health; other important considerations for this technology are equipment flexibility, low-cost components, and processing, and versatility. To meet these standards, Yamamoto proposed a flexible multifunctional printed healthcare sensor equipped with a three-axis acceleration sensor to monitor body motion and motion. Since the device is designed to be directly attached to the skin, it adopts a modular design with two removable components: one device component is non-disposable and the other is disposable, which is designed to be in contact with the skin [6]. Rathore proposed that the rapid growth of urban population density requires the provision of services and infrastructure to meet the needs of urban residents. Therefore, the increasing demand for embedded devices such as sensors, actuators, and smart phones has brought great commercial potential to the new era of the Internet of things (IOT), in which all devices can interconnect and communicate with each other through the Internet. Therefore, Internet technology provides a way to integrate and share public communication media. With this knowledge, in this paper, we propose a combined system based on the Internet of things for smart city development and urban planning using big data analysis. We propose a complete system composed of various types of sensor deployment, including smart home sensors, vehicle networks, weather and water sensors, intelligent parking sensor, and monitoring objects [7]. Internet of things (IOT) is a global infrastructure that connects objects and enables data generation and data sharing. Internet of Things is considered one of the most important fields of future technology, which has attracted great attention of researchers and practitioners in recent years. The applications presented by the Internet of Things make a large amount of developments possible, but they are rarely used at present. With the rapid development of system technology, successful implementation schemes will continue to appear to improve the quality of life in many fields. The unbalanced development of sports talent mainly occurs in the period of China's economic system transformation. Sports reform is also facing the important problem of how to make sports develop in a market-oriented way. After a series of policy support and exploration and development of sports marketization, there has been an unbalanced development of regional sports talents due to lack of experience and blindly copying the Western business model. This phenomenon has become a prominent problem in the process of China's Sports Reform [8]. The results of various scholars show that sports are becoming increasingly important in today's social development, but people do not pay enough attention to sports, so how to design action detection devices in sports based on in-depth learning of the Internet of things has become a difficult problem.

The innovation of this paper lies in the following: (1) based on the Internet, through the investigation and research method, this paper investigates and studies the three dimensions of teenagers' sports motivation, sports behavior, and sports attitude, studies and analyzes the actual effect of sports applications on college students, and then discusses the health communication effect of sports applications. (2) Using the volume accumulation algorithm, some motion detection devices are designed in sports based on the in-depth learning of the Internet of things to promote the popularization of the importance of sports. Outdoor sports motivation and sports atmosphere of adolescents are important factors affecting sports persistence. At the same time, there is a significant correlation between sports motivation, sports atmosphere, and sports persistence. The outdoor sports motivation of adolescents can directly affect the persistence of sports and can also indirectly affect the persistence of sports through the sports atmosphere. The sports atmosphere plays a significant mediating role between sports motivation and sports persistence.

## 2. Convolution Operation Based on Deep Learning of Internet of Things

### 2.1. Convolutional Neural Network

Convolutional neural network (CNN) is a multilayer neural network.  Figure 1 shows the basic architecture of the convolutional neural network [9].

As shown in Figure 1, the convolutional neural network is mainly composed of five layers: input layer, convolution layer, sampling layer, fully connection layer, and output layer. The following describes the functions of each level in details: (1) input layer: the original data enters the convolutional neural network system through the input layer. Generally speaking, when the convolutional neural network acts on image processing, the pixel value of the image can be used as direct input data. (2) Convolution layer: it is also called feature extraction layer. In the classical CNN network structure, the convolution operation is generally a classical two-dimensional convolution operation, and each convolution operation of the input image will bring changes in space size [10]. Convolution (also known as convolution) and deconvolution (also known as deconvolution) are a mathematical method of integral transformation, which has been widely used in many aspects. This layer can be used for depth extraction of shallow features of the image. (3) Sampling layer: the main function is to eliminate the irrelevant small interference that may be brought by each convolution operation and minimize the irrelevant data and its processing capacity on the basis of retaining useful information, to speed up the training network. Sampling is done independently in each depth dimension, so the depth of the image can remain unchanged. Generally speaking, common sampling operations include maximum sampling, average sampling, etc. (4) Fully connected layer: to form the final output, you need a fully connected layer to generate the output in the same number of target categories. The output layer has the same loss function as softmax that can be used to calculate the prediction error [11]. After the forward propagation is completed, the inverse propagation starts to update the weight and deviation to reduce errors and losses. Convolution is a mathematical operation. Convolution can be divided into continuous and discrete cases [12]. Their definitions are as follows.

Continuous definition:

(1) $$\begin{array}{c} \left(f*g\right)\left(n\right)=\int_{-\infty }^{+\infty }f\left(x\right)g\left(n-x\right)\text{d}x. \end{array}$$

Discrete definition:

(2) $$\begin{array}{c} \left(f*g\right)\left(n\right)=\sum_{-\infty }^{+\infty }\int_{-\infty }^{+\infty }f\left(x\right)g\left(n-x\right). \end{array}$$

The convolution operation of a convolution neural network belongs to the discrete convolution, and the size and number of convolution kernels can be flexibly defined [13]. The function of 1 *∗* 1 convolution is to linearly deform the input without affecting the input and output dimensions and then perform nonlinear processing through Relu to increase the nonlinear expression ability of the network. Generally, a small number of convolution kernels can be set in the convolution layer close to the input layer; later, the number of convolution kernels increases. After the convolution operation of two 1 *∗* 1 convolution kernels, it becomes two 2 *∗* 2 characteristic graphs, as shown in Figure 2.

### 2.2. Offline Ranking Regression Model

The offline similarity ranking regression method in this paper is based on Ndcg ranking model. The model is a classical model, which is often used as an index to measure the sorting quality [14]. NDCG (normalized loss, cumulative gain) believes that results with a high degree of relevance affect the final index score more than results with a general degree of relevance. When a result with a high degree of relevance appears in a higher position, the higher the index will be. The common formula is as follows:

(3) $$\begin{array}{c} Y=X_{M}^{-1}\times W\\ =X_{M}^{-1}\times \sum_{X\in Z}\frac{2^{R\left(X\right)}-1}{\log_{2}\left(1+\Pi \left(x\right)\right)}. \end{array}$$

*X* represents the sample block patch in the video frame; *R* (*x*) represents the area coverage ratio between the current sample block and the manually selected standard block; the area coverage between the sample block and the manually selected standard block relates to the technical field of software testing, especially to the unit test coverage generation method, device, readable storage medium, and equipment. *R* represents the position of the current sample block in the overall sorting; it is the largest normalized term in X. When the area coverage ratio of all sample blocks and standard blocks is arranged in descending order from large to small, the maximum value of *X*/*y* can be obtained, and the value range of *Y* is within [0, 1]. Although the similarity function to be learned in this article cannot be seen directly from equation (3), it can be obtained and optimized according to the ranking model. To completely introduce the offline sorting learning regression method of the whole similarity function, the following will comprehensively introduce the traditional random gradient algorithm and another more effective approximate gradient learning algorithm:

(4) $$\begin{array}{c} \pi \left(x\right)≅1+\sum_{y=x}\text{sign}\left(f\left(x,y\right)\right),\\ \pi \left(x\right)≅1+\sum_{y=x}\text{sign}\left(f\left(y\right)-\left(x\right)\right). \end{array}$$

The function is further improved, where *X* represents the function variable and *Q* controls the smoothness of the improved function. It is easy to see from formula (5) that the smaller x is, the closer the improved function is to the original Signum. In this way, the improved position function can be represented by

(5) $$\begin{array}{c} \pi^{\prime }\left(x\right)≅1+\sum_{y=x}\text{sign}\left(f\left(x+y\right)\right), \end{array}$$

(6) $$\begin{array}{c} \pi^{\prime }\left(x\right)=1+\sum_{y=x}\frac{f\left(x,y\right)}{\sqrt{f^{2}\left(x,y\right)+\alpha^{2}}}. \end{array}$$

Meanwhile, by introducing formula (5) into the *Y* model of formula (6) above, a new model formula (7) can be obtained, which is named *W*:

(7) $$\begin{array}{c} aY=N_{M}^{-1}\times \sum_{X\in Z}\frac{2^{R\left(X\right)}-1}{\text{long}\left(2+\sum_{X\in Z}\left(x-y/\sqrt{f^{2}\left(x,y\right)}\right)\right)}. \end{array}$$

Based on formula (7), a new gradient function expression can be obtained by continuously using the twice chain rule:

(8) $$\begin{array}{c} \frac{Y\left(x\right)}{\partial \theta }=N_{M}^{-1}\times \sum_{X\in Z}\frac{2^{R\left(X\right)}-1}{\log_{2}^{2}\left(1+\pi \left(x\right)\right)}. \end{array}$$

Therefore, based on the displayed gradient expression in formula (8), the end-to-end learning of the model based on SGD algorithm can be realized. Secondly, another more effective proximal gradient descent (PGD) algorithm is introduced to realize the ranking regression learning of offline similarity function [15]. The main idea is to transform the similarity learning problem into a regularization problem with lasso form, which can be expressed by the following:

(9) $$\begin{array}{c} \min\left(Z-N_{M}^{-1}\times \sum_{X\in Z}\frac{2^{R\left(X\right)}-1}{\log^{2}\left(2+\sum_{Y=Z}\left(f\left(y,x\right)/a^{2}\right)\right)}\right),\\ \min\left(Z-N_{M}^{-1}\times \underset{X\in Z}{\sum }\frac{2^{R\left(X\right)}-1}{\log^{2}\left(2+\sum_{Y=Z}\left(f\left(y,x\right)/a^{2}\right)\right)}\right). \end{array}$$

To quickly solve the above lasso problem, the proximal gradient descent (PGD) algorithm can be used. PGD algorithm is also an iterative algorithm; in each individual iteration, after the learning result *θ*_*K*−1_ is obtained from iteration *k* − 1, it is immediately sent to equation (9) to solve the intermediate variable *Q*_*K*−1_, as shown in the following:

(10) $$\begin{array}{c} Q_{K-1}=\theta_{K-1}-\frac{1}{L}\Delta F\left(\theta_{K-1}\right), \end{array}$$

where *l* represents a positive scale factor and a gradient. Here, the soft threshold idea can be used to calculate the i-th dimension of iteration *Q*_*K*−1_ in formula (10) [16], as shown in

(11) $$\begin{array}{c} \theta_{k}^{j}=\mathrm{sgn}\left(Q_{K-1}^{I}\right)-\frac{\lambda }{L}\cdot \left\{\left|Z_{K-1}^{I}\right|-\frac{\lambda }{L},0\right\}. \end{array}$$

### 2.3. Grayscale Method

The set of pixels constitutes a digital image, which can be divided into the following two categories: gray image and color images. The image directly collected by the camera is a color image [17]. In the RGB model, each color is a component image, each component image is a bit image, and each color image is composed of three component images. Due to the introduction of gray image, image processing brings a lot of convenience, the algorithm program becomes simple, and the speed of image processing is also improved. Therefore, in practical applications, color images are often output in gray. When *a* = *t* = *y*, it represents the gray color, so that the three equal values are the gray value. The following is the graying method.

#### 2.3.1. Maximum Value Method

The maximum value method is to take the largest of the three values as the values of a, *t*, and *y*, as shown in

(12) $$\begin{array}{c} A=T=Y=\max\left(A,T,Y\right). \end{array}$$

The gray image obtained by this method has high brightness.

#### 2.3.2. Average Method

The average method takes the average of the three as the values of *a*, *t*, and *y*, as shown in

(13) $$\begin{array}{c} A=T=Y=A+T+Y\left(A,T,Y\right). \end{array}$$

#### 2.3.3. Weighted Average Method

The weighted average method assigns values to a, *t*, and Y according to importance or other requirements and calculates the weighted average of the three, as shown in

(14) $$\begin{array}{c} A=T=Y=\frac{\left(W_{A}A+W_{T}T+W_{B}B\right)}{3}. \end{array}$$

### 2.4. Neighborhood Average Method

The specific operation of the neighborhood average method is to take a template and slide it on the image and then replace the pixel value at the center of the template with the average value of all pixels in the image covered by the template [18]. Let the image *g*(*a*, *b*) be an *n* × *n* array, and *w*(*a*, *b*) represents the smoothed image:

(15) $$\begin{array}{c} w\left(a,b\right)=\frac{1}{M}g\left(a,b\right). \end{array}$$

In equation (15), *a*, *b* = 0, 1, 2,… *n* − 1, *G* represents the set of neighborhood coordinate points centered on (*a*, *b*), and the range of *S* is different Including point (*a*, *b*); M represents the number of coordinate points in the *G* set. The neighborhood average method can filter out some interference. This method has a simple algorithm and a small amount of computation, but it makes the image blurred.

#### 2.4.1. Frequency Domain Low-Pass Filtering

Through the analysis of the Fourier frequency of the image, it can be seen that the slower changes of the background and image are mainly in the low frequency band, and the details, edges, and noise are mainly in the high frequency band. The noise component is filtered by the high-frequency part to obtain a smoother image [19]. Using convolution, expression (16) can be obtained.

(16) $$\begin{array}{c} T\left(u,v\right)=H\left(u,v\right)\cdot S\left(u,v\right). \end{array}$$

Here, the Fourier transform of the noisy image is represented by *S*(*u*, *v*), the Fourier transform of the smoothed image is represented by *T*(*u*, *v*), and the transfer function is represented by *H*(*u*, *v*). The high-frequency component of the noisy image is attenuated by *H*(*u*, *v*). After obtaining *T*(*u*, *v*), the desired image *S*(*u*, *v*) is obtained by inverse Fourier transform.

#### 2.4.2. Median Filtering

If the window has 5 points whose values are 70, 80, 140, 90, and 120, the median value of each point of the window is 90, and 90 is assigned to the center point of the window. Suppose *q*_1_*q*_2_ … *q*_*n*_ represents a one-dimensional sequence. Assuming that the window length is *m* (*M* is an odd number), median filtering is performed on the sequence. In other words, *m* values are taken out in sequence from *q*_*i*−*v*_*q*_2*i*−1_*q*_*i*_*q*_*i*+1_ … *q*_*i*+*v*_ input, and M points are listed according to this value. This represents the center value of the window, and the middle value is used as the output of the filter, as shown in

(17) $$\begin{array}{c} Y_{I}=\left\{q_{i-v}q_{2i-1}q_{i}q_{i+1}\ldots q_{i+v}\right\}. \end{array}$$

### 2.5. Background Subtraction

The most commonly used moving target detection algorithm is background subtraction to detect moving targets by subtracting the current frame image and background image [20]. Background subtraction has the advantages of less computation, easy implementation, high anti-interference ability, and obtaining the complete information characteristics of the moving target. Therefore, the moving target can be segmented appropriately from the video image. Therefore, many researchers often use this method for moving target detection [21]. Assuming that *f*_*k*_ represents the current frame image, B represents the background image, and *T*_*k*_ represents the subtracted image, the subtracted image is shown in

(18) $$\begin{array}{c} T_{k}\left(x,y\right)=f_{k}\left(x,y\right)-B_{k}\left(x,y\right). \end{array}$$

As shown in Figure 3, when using background subtraction, the camera needs to be fixed. Generally speaking, the background image sequence follows Gaussian distribution, and the noise is almost white noise. Whether the background template is properly selected plays a vital role in the accuracy of the background subtraction method. Now many researchers are committed to developing different background templates to make the detection more accurate. The background subtraction method is an effective moving object detection algorithm. The basic idea is to use the parameter model of the background to approximate the pixel value of the background image and compare the current frame with the background image to achieve the detection of the moving area. The difference is larger. The pixel area is regarded as the motion area, and the pixel area with smaller difference is regarded as the background area [22].

### 2.6. Infrastructure of “Two Bridges and Two Foundations” Communication System

The theoretical structure of “two bridges” in the “two bridges, two foundations” communication system is two forms of communication: talent market and sports broker. Although they both have the function of communication, there are essential differences and characteristics between them [23]. The basic structure of the communication system is the signal generation part plus the signal sending system. Modern communication systems are mainly realized by the propagation of electromagnetic waves in free space or the transmission mechanism in the guiding medium. The talent market and sports brokers are the products of China's economic system transformation. The talent market has built a platform for China's talent exchange in the new era. The talent market has played its own unique role as a fixed exchange platform and provided a communication place for negotiation and communication between the supply and demand sides. Sports brokers provide communication and intermediaries for athletes and sports institutions in the process of sports market development. Sports brokers have their own special mobile communication platform in the communication system. Through the successful commercialization of sports agents, many athletes seek a suitable sports development space. Mastering the two forms of communication is of great significance to athletes' communication in the new era, as shown in Figure 4.

At present, China's sports medical industry has a lack of talent, people also lack understanding of sports medical treatment, and the market of the combination of sports medical treatment in China is blank. In the 13th five-year plan for youth sports released by the state in September 2016, it was advocated to track users' sports data and body data through sports applications and provide sports medical services through intelligent analysis of sports big data [24]. Airy Consulting and Reporting Center has made a preliminary investigation on the route of combining sports and medicine, as shown in Figure 5.

It can be seen from Figure 5 that sports applications should be good at giving full play to their own advantage, combining sports and medical treatment with big data, so that users can get corresponding health services while exercising.

The Internet of things is a network system that gives things related to human activities, the ability to perceive or be perceived, through the collection and processing of information, group embedding, identification, network transmission, arrangement and services to humans, and making human production and life more intelligent and efficient. The Internet of things technology has several trend characteristics, such as comprehensive perception, ubiquitous interconnection, and intelligent mining.  Figure 6 is a structural diagram of the Internet of things.

## 3. Experiment and Analysis

### 3.1. Experiment and Analysis of Questionnaire Survey Method

Deep learning is to learn the internal laws and representation levels of sample data. The information obtained in the learning process is of great help to the interpretation of data such as text, images, and sounds. Its ultimate goal is to allow machines to have the ability to analyze and learn like humans, and to recognize data such as text, images, and sounds. Questionnaire survey is widely used in social surveys at home and abroad. Questionnaire survey refers to the form of statistics and survey in which questions are expressed by asking questions. According to the research content requirements of this paper, the authors designed a questionnaire for the research problems. To ensure the scientificity and effectiveness of the questionnaire, it was repeatedly modified on the basis of previous personal interviews and distributed after preliminary prediction tests and analyzed the user experience, usage, and other data of sports applications; several cases are selected from the students who use it frequently for in-depth interviews to enrich the demonstration. The questionnaire method is to use properly designed questionnaire tools for investigation. Because the design of the questionnaire needs standardization and measurement, it provides data support for discussion. Because China did not fully analyze the related problems, such as the poor foundation of its sports market, regional environmental differences, lack of reform experience, and blindly copying foreign models, a series of athlete exchange problems appeared in the transition period. At present, in view of various adverse phenomena in China's sports transformation period, it is an effective method to determine the main factors behind the phenomenon through scientific analysis and determine reasonable solutions through systematic research. (1) Development status of sports applications since 2017: the sports application market has gradually presented a “blue ocean” landscape. According to the National Fitness plan (2016–2020) issued by the State Council, the output value of China's fitness industry was 146.5 billion yuan in 2016 and 167 billion yuan in 2019, showing a linear growth and scale development, as shown in Figure 7.

As can be seen from Figure 7, from 2016 to 2018, the market entered a period of rapid growth, and various sports applications mushroomed, showing a “blowout” development until 2019. On the whole, the current overall development of sports applications gradually tends to be mature, the revenue scale increases rapidly, and the user group tends to be stable. With the trend of sharing economy, shared fitness has become a new trend in the future.

#### 3.1.1. Questionnaire Design and Research Framework

The number of sample data and the validity of a single questionnaire are the basis for the validity of the questionnaire. When designing the questionnaire from the standpoint of the respondent, when considering and designing for them, the questionnaire can be effectively retrieved to a large extent. Based on the theory of emotional design, the theory of planned behavior, and the model of knowledge, belief, and behavior, combined with the partial adjustment and revision of the Chinese college students' physical exercise behavior change scale, and the interview with the previous survey objects, this paper constructs the research model of this paper and puts forward some hypotheses. According to the calculation formula of sample size, the college students are investigated at the 95% confidence level (*t* = 1.96), and the minimum sample size under this condition should be between 100 and 300. Considering that invalid samples may appear in the actual questionnaire survey, the sample number of this study is initially determined as 350. Due to the characteristics of the research object, the sampling method adopted in this study is non-random sampling. Before the formal distribution of the questionnaire, the authors conducted a pretest within the WeChat group chart in the dormitory building and distributed 30 questionnaires, 21 of which were valid. After the prediction questionnaire is collected, the reliability of the collected results is tested. In this study, Cronbach's alpha was used and the internal consistency of the two scales was analyzed. Due to the setting of the “questionnaire star” interface, the scores of some matrix quantization tables are substandard, so some adjustments and modifications are made to the questionnaire after synthesis. The modified Cronbach of the two scales *α* is shown in Table 1. Cronbach's coefficient is a statistic, which refers to the average of the half-reliability coefficients obtained by all possible item division methods of the scale, and is the most commonly used reliability measurement method. Cronbach values of the two scales are between 0.75 and 0.77, indicating that the reliability of Table 1 is acceptable.

It can be seen from Table 1 that the Cronbach *α* value can represent the relationship between user experience perception and health perception, because its values are all above 0.75, so it can affect sports behavior. The questionnaire is filled in anonymously and distributed online and offline. It can be seen from Table 1 that sports applications mainly affect sports behavior through user experience, cognition, and health cognition presentation, and then affect the establishment of users' health beliefs. The establishment of users' health beliefs will also affect users' sports behavior in turn, so that their health has been improved imperceptibly.

#### 3.1.2. Gender Structure and Education Level

Sports applications are not only the media, but also an attitude towards life. Many studies have shown that many users take the initiative to search when downloading and using applications, which subconsciously strengthens the dissemination of youth subculture to some extent, and a healthy culture that promotes sports and physical fitness also spreads, expanding the connotation and extension of sports. Therefore, some sports applications will have the words “healthy life” on the user interface to give users psychological hints. Therefore, through the investigation of different genders of undergraduates and masters, we get Figure 8.

Figure 8, after cross analysis, in this questionnaire, about 39.8% of male students and 60.2% of female students are willing to participate in sports. In terms of educational background, after cross-analysis between gender and education level and whether to use sports applications, about 24.32% of male students use sports applications, and about 75.58% of female students use sports applications. Students with a master's degree or above may be more willing to use sports applications because there are few undergraduate students in the course. However, it can be predicted that even if comprehensive data protection laws are issued, whether foreign or domestic, it may not be able to deal with all practical problems. New problems will continue to emerge in the information society and intelligent society, and the contradiction between data governance and privacy protection will exist for a long time, but no matter how the problem changes, some basic principles should be followed.

As shown in Figure 9, after cross-analysis, in this questionnaire, the number of boys willing to exercise from 2016 to 2017 increased by about 12%, and the number of girls by about 16%. By 2020, boys' willingness to participate in sports will increase to 35%, and girls' willingness to participate in sports will increase to 36%. This shows that, regardless of men and women, interest in sports is increasing year by year, so sports should be paid more attention to.

This paper proposes a wearable student physical fitness monitoring system based on ARM embedded technology, which is used to monitor physical parameters such as body temperature and heart rate during physical exercise of students and upload the data to the cloud service center for data monitoring, in addition to analysis to prevent accidents such as fainting and death when students exercise.

### 3.2. Experiment and Analysis of Quantitative Method

Through the investigation of students in a university, it is found that most of them think they are in a subhealth state and generally agree that physical exercise is particularly useful for their own physical health, but they know that the reason for subhealth is their lack of physical exercise.

It can be seen from Table 2 that more than 50% of college students have a strong interest in sports and fitness, but the actual situation is less than 30%, which is not optimistic. There are many reasons for college students' slack exercise, such as weak willpower and inability to concentrate. In terms of sports applications designed for college students, we should pay more attention to enhancing the stickiness of college students. We can not only use some “cash” rewards, but also jointly launch some physical objects or activities closely related to our students' daily campus life to promote college students to participate in sports and exercise.

Body-wearable fall detection systems usually use airborne inertial sensors, such as three-axis accelerometers and gyroscopes. The combination of features derived from these signals is used to detect whether a fall occurs at any given moment. Optionally, other sensors such as pressure sensors can be used to detect changes in height.

## 4. Discussion

This paper analyzes the design of motion detection devices in sports based on Internet of things deep learning, expounds the concepts related to Internet of things deep learning and sports, studies the relevant theories based on Internet of things deep learning, explores the design method of motion detection devices in sports, and discusses the importance of sports to contemporary society through questionnaire cases. Finally, it takes the integration of the Internet into sports as an example to explore the correlation between the two.

This paper also makes rational use of convolution operation based on deep learning of Internet of things. With the increasing application scope and the importance of data fusion, many scholars have begun to match some specific fusion theories with real application scenarios and put forward feasible algorithms. Convolution is a mathematical operation. Generally, the convolution can be expressed in the form of. Convolution can be divided into continuous and discrete cases. According to the calculation, strengthening sports activities through the Internet is an essential part of life.

Through the questionnaire survey, we can know that the teaching process of the traditional college physical education classroom is too single and lacks interest. The survey data of this paper also shows that most students have sports enthusiasm and demand cognition, but they are unwilling to participate due to willpower and other reasons. During the physical fitness test, the setting of the online “sports scene” makes the “frightening” physical fitness test become an interesting competition among students. It is combined with sports applications to investigate students' exercise volume and usual performance, which not only improves teachers' classroom efficiency, but also increases teachers' personality charm and stimulates the relationship between teachers and students.

## 5. Conclusions

The suggestion of this article is to increase investment in physical education, purchase necessary sports goods and equipment for schools, and establish and improve the management system for the maintenance and use of sports facilities and sports equipment. Starting from the Internet deep learning and sports, this paper discusses the relationship between the two and how to design the action detection device in sports based on the Internet of things deep learning. The volume calculation based on the Internet deep learning can be learned: with the strong encouragement of the state and everyone's attention to physical health, sports application products effectively combine the Internet with sports and fitness in development. Online platform combines Internet plus sports fitness to attract users to participate in sports through abundant communication strategies such as sports data visualization. Online combination of sports fitness and Internet can greatly improve people's interest and practicality in sports. There are a wide range of scientific fields related to the design of motion detection devices in sports with in-depth learning of the Internet of things. Sensors have the potential to improve athletic ability, balance the competitive landscape, create fair referees, and increase fan interaction. Understanding how sensors are changing today's sports and their potential future impact can enhance the interest of the remaining 70% of students in sports. There has always been a dispute over the concept of sports. The authors' academic knowledge is still relatively weak, so it is inevitable that there are deficiencies. There are still some problems in the design work. At the same time, the authors are also constantly discovering and solving problems, hoping to do better.

## Figures and Tables

**Figure 1:** Basic structure diagram of convolutional neural network (CNN).

**Figure 2:** Schematic diagram of convolution operation.

**Figure 3:** Flow chart of background subtraction method.

**Figure 4:** Pictures of athletes in the new era.

**Figure 5:** Imports to medical treatment.

**Figure 6:** The structure diagram of the internet of things.

**Figure 7:** Statistical chart of output value of China's fitness industry.

**Figure 8:** Bar chart of percentages by gender and educational background.

**Figure 9:** Combination diagram of men and women attaching importance to sports year by year.

**Table 1:** Cronbach's alpha scale.

	Cronbach's alpha	Cronbach's alpha *α*	Number of items
User experience perception	0.765	0.782	7
Health perception	0.752	0.773	3

**Table 2:** Health questionnaire.

Object	Grade	Self-evaluation (%)	Usage frequency (%)	Whether to follow (%)	Whether to exercise (%)
A	Girl	45	57	26	12
B	Boy	50	77	15	18
C	Girl	53	75	19	23
D	Boy	46	86	21	16
E	Girl	48	67	16	21
F	Boy	38	76	12	26
G	Girl	37	57	20	15
H	Boy	42	78	22	20
I	Girl	47	73	17	17
J	Boy	39	85	18	19

## Data Availability

Data sharing is not applicable to this article as no datasets were generated or analyzed during the current study.
